# Computational design and molecular modeling of the interaction of nicotinic acid hydrazide nickel-based complexes with H_2_S gas†

This article has been retracted.

**DOI:** 10.1039/d2ra05456f

**Published:** 2022-10-24

**Authors:** Hitler Louis, Daniel Etiese, Tomsmith O. Unimuke, Aniekan E. Owen, Abdulahi O. Rajee, Terkumbur E. Gber, Chioma M. Chima, Ededet A. Eno, Emmanuel N. Nfor

**Affiliations:** Computational and Bio-Simulation Research Group, University of Calabar Calabar Nigeria louismuzong@gmail.com; Department of Pure and Applied Chemistry, Faculty of Physical Sciences, University of Calabar Calabar Nigeria; Department of Chemistry, Akwa-Ibom State University Uyo Nigeria; Department of Chemistry, University of Ilorin Ilorin Nigeria; Department of Chemistry, University of Buea Buea Cameroon

## Abstract

The application of nickel complexes of nicotinic acid hydrazide ligand as a potential gas-sensor and adsorbent material for H_2_S gas was examined using appropriate density functional theory (DFT) calculations with the ωB97XD/Gen/6-311++G(d,p)/LanL2DZ method. The FT-IR spectrum of the synthesized ligand exhibited a medium band at 3178 cm^−1^ attributed to *ν*(NH) stretching vibrations and strong bands at 1657 and 1600 cm^−1^ corresponding to the presence of *ν*(C=O) and *ν*(C=N) vibration modes. In the spectrum of the nickel(ii) complex, the *ν*(C=O) and *ν*(C=N) vibration bands experience negative shifts to 1605 cm^−1^ and 1580 cm^−1^, respectively, compared to the ligand. This indicates the coordination of the carbonyl oxygen and the azomethine nitrogen atoms to the Ni^2+^ ion. Thus, the sensing mechanism of the complexes indicated a short recovery time and that the work function value increases for all complexes, necessitating an excellent H_2_S gas sensor material. Thus, a profound assertion was given that the complex sensor surfaces exhibited very dense stability with regards to their relevant binding energies corresponding to various existing studies.

## Abstract 2

We demonstrate the efficacy of nicotinic acid hydrazide as adsorbent/sensor materials for H_2_S gas.

## 1. Introduction

Hydrogen sulphide (H_2_S) from natural and anthropogenic sources is a highly irritating, flammable, acutely toxic, and extremely hazardous and corrosive gas that must be captured and removed from several important gaseous and liquid streams.^1^ The concentrations in ambient air range from 0.11–0.33 ppb and in urban areas are generally <1 ppb, although much higher concentrations (often exceeding 90 ppb) have been detected in certain communities.^2^ According to the Occupational Safety and Health Administration and the Bureau of Labour Statistics, H_2_S is one of the most dangerous gases in occupational settings.^3^ Long and acute exposure to high levels of H_2_S is known to elicit several organ toxicities including neurotoxicity, chronic respiratory failure, and even, in other unattended, and/or serious cases, death.^4–6^ As a result of its serious harmful impacts on humans, ecological environment and social economy, the capture, conversion and removal of this compound from these streams has become imperative.^7^

Gas chromatography or spectrometry are some common analytical methods used to quantify H_2_S concentration in air. Many drawbacks are presented such as complex sampling and analyzing processes, high cost, and low temporal resolution or posterior measurements in a case where hydrogen sulphide possesses a considerable high sensitivity toward low concentration.^8,9^ Effective measures for odour monitoring and safety control require user-friendly, cost-effective and continuous real-time measurements. Many researchers have worked on developing swift, portable, and low-cost devices, in the absence of standardized methods for satisfying those requirements.^10^ Chemoresistive, electrochemical, and optical sensors are notable popular devices developed for H_2_S sensing.^11,12^ The sensitivity and stability of sensors still need to be optimized, even if few have been commercialized. This established challenge has given rise to different technologies emanating from different types of materials over the years.^1^

There is a growing need for fast and efficient detection of toxic gases and cancer biomarkers^13,14^ due to the strict limits on food safety, indoor air quality monitoring, emission control, medical diagnosis and public security.^15^ Sensing materials which can concentrate and adsorb gases onto the surface of the sensors, and then generate a signal for detection play a vital role in detecting gases. Gas sensors are tools for detecting various gases, and they should cater for several requirements, including high sensitivity operation, low limit-of-detection (LOD), and long-term stability. In order to meet the challenges in the design of gas sensors, materials such as carbon-based nanomaterials,^16^ metal oxide semiconductors (MOSs),^17^ conductive polymers,^18^ solid electrolytes,^19^ and some two-dimensional nanostructured materials have been explored.^20,21^ Organic and carbon-based materials usually show poor stability and not enough sensitivity. Contrastively, inorganic materials, such as MOSs, operate at significantly high temperatures, resulting in baseline drift and oxidation of analytes. These pitfalls hinder the development of gas sensors.^22^ Owing to these, it is imperative to develop gas sensors with high sensitivity for real-time monitoring of H_2_S.

Recently, metal–semiconductor materials have been introduced owing to their excellent properties and have shown promising potential to detect H_2_S gas.^23^ Among these materials, the inorganic tungsten oxide (WO_3_) nanoparticles have been noted across fields to have the potential for practical applications.^24^ Similarly, other sensors containing iron, cadmium, copper and indium oxides were found to be selective toward H_2_S detection in ppm concentration levels.^25–28^ At very low levels, both ZnO and TeO_2_ films were found to be highly sensitive to H_2_S gas.^29^ The design and use of metal complexes for H_2_S gas detection would help achieve the optimum enhancement of H_2_S sensors in terms of sensitivity, selectivity, and rapid response^30^ as varying the central metal ion is an effective tool to govern the sensitivity and selectivity of these compounds, as the metal next to the substituents is known to largely influence the sensing properties.^31^ Among the transition metal oxides, nickel oxide has attracted much attention due to its properties and applications.^32^ While the vast majority of research works on the application of metal complexes as sensors has been devoted to biological systems,^33–35^ there has been limited research progress on environmental gas sensing properties. Hence, this research work is focused on the synthesis, characterization, and the theoretical modelling of the gas (H_2_S) sensing properties of nickel complexes of nicotinic acid hydrazide ligand.

## 2. Methods

### 2.1 Experimental

#### 2.1.1 Synthesis of the ligand

Nicotinic acid hydrazide (0.27 g, 2 mmol) was added to indole-3-carboxaldehyde (0.29 g, 2 mmol) in 25 mL of ethanolic solution with three drops of glacial acetic acid added as catalyst. The resulting mixture was refluxed for five hours at a temperature of 70 °C with continuous stirring. The product was left to cool overnight, and removed by vacuum filtration; the product was washed several times with water, ethanol, and diethyl ether and dried in a desiccator. Yellow crystals suitable for single crystal X-ray diffraction studies were obtained from the ethanolic filtrate after 30 days.^36^

#### 2.1.2 Synthesis of the metal complex

The Schiff base, L_1_, (0.26 g, 0.5 mmol) was added to Zn(CH_3_OO^−^)_2_·2H_2_O (0.046 g, 0.25 mmol) in a 25 mL ethanolic solution. The resulting mixture was refluxed for 5 hours at a temperature of 80 °C with continuous stirring using a magnetic stirrer. The pale-yellow solution obtained was allowed to cool overnight, the products removed by filtration; washed with ethanol and stored in a desiccator.^36^

#### 2.1.3 X-ray crystallography

Orange single crystals (plate-like with 0.952 × 0.685 × 0.264 mm^3^ for L_2_) was served for analysis. The samples were set on top of a glass capillary, coated with a thin layer of Araldite epoxy resin. Intensity data were collected on a Bruker APEX2 CCD diffractometer (Bruker, Billerica, MA, USA) with Mo-Kα radiation monochromated by graphite (*λ* = 0.71073 Å) at 173.2 K. Data treatment used the program package SAINT (Bruker, Billerica, MA, USA). An empirical absorption correction for intensity was applied by the program SADABS (Bruker, Billerica, MA, USA). In this program package, the structures (phase problem) were initially solved by direct methods with a SHELXS-97,^22^ expanded by Fourier techniques, and finally refined by full-matrix least-squares methods based on *F*^2^ using a SHELXL-97 program.^22^ All non-hydrogen (heavy) atoms were readily located to construct a model and were refined by anisotropic (thermal) displacement parameters. Hydrogen atoms were located at geometrically calculated positions and refined using riding models.^36^

#### 2.1.4 IR spectroscopic characterization

The infrared spectra of the ligand L_1_ and its metal(ii) complexes were recorded within the 4000–400 cm^−1^ region using the Fourier-transform infrared spectrometer Thermo scientific NICOLET 6700 equipped with an MCT detector. The spectrum consisted of an accumulation of 16 scans obtained at a resolution of 4 cm^−1^. The instrument was connected to an Omnic software, which extended from 400 to 4000 cm^−1^.^36^

### 2.2 Computational details

In this work, ground state geometrical optimizations, for all the studied systems, were carried out within the framework of DFT with the help of Gaussian 16 programs.^37,38^ The ground state energy of all the systems was optimized in a vacuum using the GEN method by assigning the 6-311++G(d, p) and LanL2DZ for lighter (C, H, N, O) and heavy (nickel) atom respectively. The hybrid long-range separated empirical-corrected dispersion, ωB97X-D functional developed by Head-Gordon *et al.*^39^ was chosen for the complete calculations. Reactivity, stability and electronic charge distribution utilizing the highest occupied molecular orbital and lowest unoccupied molecular orbital (HOMO–LUMO) were computed at DFT/ωB97XD with 6-311++G(d,p) to investigate the reactivity and stability of the modelled compounds. The plots of the HOMO–LUMOs were plotted by utilizing the checkpoint file from the optimized structure to study the distribution of electrons. By invoking Gaussian 16, natural bond orbital (NBO) analysis that utilizes the stabilization energy to study the magnitude of inter and intramolecular charge transfer between molecules was computed using the in-built Gaussian 3.1 methods available in Gaussian 16 software. GaussSum and Multiwfn 3.7 software were used to plot the PDOS.^40,41^ To gain deeper insight into the nature of the interatomic interactions, the topological analysis – quantum theory of atoms in molecules (QTAIM)^42^ and noncovalent interaction (NCI) isosurface maps investigations were extracted by Visual Molecular Dynamic (VMD) 1.9.3 program^43^ based on the outputs of Multiwfn analyzer. Adsorption energy involved during the adsorption of the gas on the complexes was calculated using eqn (1) (ref. 44 and 45)

1 *E*_ads_ = *E*_complex/gas_ − *E*_complex_ − *E*_gas_ + *E*_(BSSE)_ + *E*_(ZPE)_

where *E*_complex/gas_ depicts the energy of the adsorbed H_2_S and complex, *E*_gas_, and *E*_complex_ represent the energy of the H_2_S and isolated complex individually, and *E*_(ZPE)_ as the zero-point energies of the respective studied systems.

The counterpoise approach established by Boys and Bernardi was used to determine the basis set superposition error (BSSE), which is indicated in eqn (2);^46,47^

2 Δ*E*_(BSSE)_ = Δ*E*_system_ − Δ*E*^system^_complex_ − Δ*E*^system^_gas_

## 3. Results and discussion

### 3.1 Spectroscopic characterization

The infrared spectra of the primary ligand and its nickel(ii) complex were recorded within the 4000–400 cm^−1^ region. IR spectrum of the ligand exhibited a medium band at 3178 cm^−1^ attributed to *ν*(NH) stretching vibrations. The strong bands at 1657 and 1600 cm^−1^ in the spectrum of the ligand, correspond to the presence of *ν*(C=O) and *ν*(C=N) vibration modes.^48^ Bands appearing at 995, 939, 800, and 781 cm^−1^ in the spectrum of the ligand are the usual modes of C–H of the aromatic ring vibrations and these revealed small shifts in the nickel(ii) complex compared to the ligand, which is the expected electronic structure changes that occur with coordination of the ligand to Ni^2+^ ions. In the spectrum of the nickel(ii) complex, the *ν*(C=O) and *ν*(C=N) vibration bands experience negative shifts to 1605 cm^−1^ and 1580 cm^−1^, respectively, compared to the ligand. This indicates the coordination of the carbonyl oxygen and the azomethine nitrogen atoms to the Ni^2+^ ion. In the low-frequency region, the bands in the region 520 and 492 cm^−1^ are probably due to *ν*(Cu–O) and *ν*(Cu–N) vibrations, respectively. More details on the spectroscopic characterisation of the ligand and complex is reported in the ESI.†

From the table of experimental and theoretical FT-IR data computed in Table 1, it is seen that there are four functional groups for the ligand and the complex. In this study, experimental values analyzing the spectral absorption of strong intensity around 3178 cm^−1^ correspond to the N–H stretching absorptions for the ligand which was theoretically calculated as 3361 cm^−1^. The characteristic band of strong intensity experimentally observed for the stretching vibration of C–H for the ligand was 995, 939, 800, and 781 which was theoretically calculated as 898, 792, 739, and 734 cm^−1^. The carbonyl group within the studied compounds were observed due to the non-linearity of the hydrogen bond. From the experiment, the stretching vibration corresponding to the C–O bond was observed to be 1657 cm^−1^ and 1605 cm^−1^ experimentally for the ligand and complexes and 1671 and 1623 cm^−1^ theoretically. C–N stretching vibrations are expected to be within the region 1727 cm^−1^ and 1545 cm^−1^ whereas in this work experimental values are 1600 cm^−1^ and 1580 cm^−1^. In the complex, Ni–O stretching absorptions were observed and reported as 520 cm^−1^ and 510 cm^−1^ for experimental and theoretical respectively, while Ni–N vibrations were observed at 492 cm^−1^ experimentally and at 446 cm^−1^ theoretically.

**Table 1:** Experimental and theoretical FT-IR

Structures	Experimental frequency (cm^−1^)	Theoretical frequency (cm^−1^)	Scaled frequencies (cm^−1^)	Assignment
Ligand	3178	3576	3361	*ν*(NH)
	1657	1788	1671	*ν*(C=O)
	1600	1727	1623	*ν*(C=N)
	995, 939, 800, and 781	956, 843, and 786	898, 792, 739, and 734	*ν*(C–H)
Complex	1605	1634	1535	*ν*(C=O)
	1580	1545	1452	*ν*(C=N)
	520	510	479	*ν*(Ni–O)
	492	446	419	*ν*(Ni–N)

### 3.2 X-ray crystallography and Hirshfeld analysis

The asymmetric unit of L_1_ along with the atomic numbering scheme is depicted in Fig. 2 while the modelled scheme is presented in Fig. 1. The crystal structure refinement data for L_1_ is given in Table 2. The L_1_ has two independent molecules having different torsion angle in the asymmetric unit of the crystal designated as molecule A (green) with a planar structure, molecule B (blue) with a twisted structure. There are a total of 8 molecules of C_15_H_12_N_4_O in the unit cell. The Schiff base L_1_ crystallizes in the monoclinic system in space group *P*2_1_/*c*. In L_1_, the bond distance C(21)–O(2) is equal to 1.236(3) Å indicating its double bond nature. The bond lengths N(6)–N(7) and C(21)–N(6) are equal to 1.392(3) Å and 1.342(3) Å, respectively. These bonds were however theoretically calculated to be 1.2126 Å, 1.347 Å, 1.2808 Å, 1.3828 Å respectively. The C(21)–N(6)–N(7) bond angle is equal to 120.63(17) and computationally calculated as 123.7°. Most of bond distances and angles were within common ranges of normal covalent bonds. The intermolecular hydrogen bond between (indole) N4–H⋯O1 (carbonyl) was observed for L_1_ molecule. The 6-membered aromatic rings are stacked *via* weak Π-interaction, and stacked rings of B are perpendicular to C=N bond of A.

**Fig. 1:** Optimized geometry of the studied complexes at the DFT/ωB97XD/6-311++G(d,p) level.

**Fig. 2:** Molecular structure with atom numbering scheme (b) crystal packing of distinguished crystallographic independent molecules (A = green, B = blue) and molecular structures of for L_1_.

**Table 2:** Reactivity parameters for the complexes calculated at DFT/ωB97XD/gen level of theory

Structures	*E*_HOMO_	*E*_LUMO_	Energy gap	*E*_INT_
L_1_Ni	−13.8860	−6.8712	7.0148	−37483.6146
L_2_Ni	−13.8182	−6.7854	7.0328	−35449.0141
L_3_Ni	−13.7899	−6.8178	6.9721	10 530.4520
L_4_Ni	−13.1205	−9.8707	3.2498	48 282.8089

#### 3.2.1 Hirshfeld surface analysis

Crystal Explorer 17.5 was utilized for the Hirshfeld surface analysis (HAS) to fully grasp the intermolecular interactions pertinent within L_1_.^23^Fig. 3(a) and (b), depict the predicted Hirshfeld surfaces for L_1_. The left figures show 3D Hirshfeld surfaces with intramolecular mutual constellation. Red indicates a short intermolecular distance, while blue indicates a large intermolecular distance on the de (distance from the surface to the outermost nucleus) and di (distance from the surface to the inner nearest nucleus) surfaces shown in Fig. 3. 2D fingerprint plots are shown in the right figures. The blue area denotes locations where a particular reciprocal interaction may occur. The entire plot is represented by the gray region. For L_1_, the atom–atom percent interactions between the A's (aliphatic) N–H and O=C(carbonyl) are as follows: H–H = 39.2%, H–O = 8.2%, O–H = 5.7%, N–H = 9.5%, and N–C = 6.2%, whereas the B's (aliphatic) N–H and proton donors (aromatic) tend to interact strongly with H–H = 34.2%, and H–O = 6.4% respectively.

**Fig. 3:** Hirshfeld surface fingerprint plots for the molecule L_1_ (a) A and (b) B.

### 3.3 Reactivity of hydrazide derivatives

The synthesized hydroxide obtained was further modelled into three derivatives shown in Fig. 1. The modelled ligand was co-named L_2_, L_3_, and L_4_. These ligands differ from the primary ligand by the geometry arrangement and atoms configuration. The oxygen hetero-atom in the furanic ring of the primary ligand was replaced with sulfur atoms in L_2_ making it have two thiophene rings. L_3_ also differ from the primary ligand in that one of the furanic rings was replaced with a thiophene ring. In L_4_ one of the furanic oxygen atoms from the furanic ring was replaced with a nitrogen hetero-atom bringing about two separate rings, the thiophene and pyridine ring respectively.

The energy gaps of the complexes were determined by taking the negative difference between the HOMO and LUMO. The energy gap helps to elucidate the stability of a chemical system, a lesser energy difference between the HOMO and the LUMO is indicative of less chemical stability and easier transition of electrons from the HOMO to the LUMO while a wider energy gap reflects more chemical stability which affects the ease with which electrons are transferred from the HOMO to LUMO. As seen in Table 2, L_2_Ni has the highest energy gap value of 7.0328 eV and is considered to be the most stable complex while L_4_Ni which has an energy gap value of 3.2498 eV is considered to be the most reactive complex. In order of reactivity, the complexes follow the trend L_4_Ni > L_3_Ni > L_1_Ni > L_2_Ni.

The interaction energy, *E*_INT_, is the energy contribution from each specie that forms a larger chemical specie. The interaction energy helps to determine how reactive and stable a specie is. Large *E*_INT_ values indicate more reaction between the species forming the chemical specie. From Table 2, L_4_Ni and L_3_Ni have positive interaction energy this shows that the bond between the ligands and the metal is a strong interaction while L_2_Ni and L_1_Ni values of interaction energy are negative and it's indicative of less interaction between the ligands and the metal. From the similarity, in the energy gap and interaction energy, it can be concluded that L_4_Ni is the most reactive modelled complex.

### 3.4 HOMO–LUMO analysis

The most important orbitals in a molecule are the highest occupied molecular orbital (HOMO) and the lowest unoccupied molecular orbital (LUMO), also known as frontier molecular orbitals. These orbitals give information about the molecules' electrical, optical, and reactive properties. The energies of these orbitals are used to determine quantum descriptors such as chemical potential (*μ*), chemical hardness (*η*), chemical softness (*σ*), electrophilicity (*ω*), electronegativity (*χ*), ionization potential (*I*) and electron affinity (*A*) of the studied structures using Koopmans' approximation^49^ and are displayed in Table 3. The HOMO–LUMO plots of these structures are given in Fig. 4.

**Table 3:** Quantum descriptors for the systems under study calculated at DFT/ωB97XD/gen level of theory

Structures	*I* = −*E*_HOMO_	*A* = −*E*_LUMO_	*E*_g_	*μ*	*Η*	*σ*	*ω*	*χ*
L_1_	8.1980	0.1235	8.0745	−4.1608	4.0373	0.1239	2.1440	4.1608
L_2_	8.3768	0.3230	8.0538	−4.3499	4.0269	0.1242	2.3494	4.3499
L_3_	8.3523	0.2667	8.0856	−4.3095	4.0428	0.1237	2.2969	4.3095
L_4_	3.1154	2.6874	0.4280	−2.9014	0.2140	2.3365	19.6685	2.9014
L_1_Ni	13.8860	6.8712	7.0148	−10.3786	3.5074	0.1426	15.3554	10.3786
L_2_Ni	13.8182	6.7854	7.0328	−10.3018	3.5164	0.1422	15.0903	10.3018
L_3_Ni	13.7899	6.8178	6.9721	−10.3039	3.4861	0.1434	15.2277	10.3039
L_4_Ni	13.1205	9.8707	3.2498	−11.4956	1.6249	0.3077	40.6637	11.4956
L_1_Ni–H_2_S	13.7943	6.6448	7.1495	−10.2196	3.5748	0.1399	14.6079	10.2196
L_2_Ni–H_2_S	13.7330	6.5528	7.1802	−10.1429	3.5901	0.1393	14.3281	10.1429
L_3_Ni–H_2_S	13.7048	6.5892	7.1156	−10.1470	3.5578	0.1405	14.4698	10.1470
L_4_Ni–H_2_S	13.0250	9.6048	3.4202	−11.3149	1.7101	0.2924	37.4326	11.3149

**Fig. 4:** Localization of HOMO and LUMO molecular orbitals of the studied complexes.

### 3.5 Global reactivity parameters

The chemical hardness (*η*) and softness (*σ*) of the studied systems were determined using eqn (3) and (4):34

The hardness or softness of a chemical specie could also be determined using the energy gap values. Species with large energy gaps are chemically hard species while those with smaller energy gaps are soft species and these show the degree of stability and reactivity of the specie respectively. The hardness of L_1_, L_2_, and L_3_ was observed to decrease on complexation with Ni whereas that of L_4_ increased but its value was not as high as those of L_1_Ni, L_2_Ni, and L_3_Ni. On adsorption of H_2_S on the complex, the hardness of all the complexes was observed to increase but that of L_4_Ni–H_2_S was the lowest. From this it confirms that the order of reactivity of our complex with H_2_S follows the trend L_4_Ni > L_3_Ni > L_1_Ni > L_2_Ni.

Ionization potential (*I*) is the amount of energy required to remove an electron from the surface of a chemical species, it entails the loss of an electron from a chemical specie while electronegativity (*χ*) is the measure of the ability of specie to draw electrons to itself. As can be seen in Table 3, the electronegativity of L_1_, L_2_, L_3_, and L_4_ increased on complexation with Ni. And on adsorption of H_2_S by the complexes, their electronegativity increased. L_4_Ni was seen to have the highest electronegativity before and after adsorbing H_2_S.

### 3.6 Natural bond orbital (NBO) analysis

The charge distribution between the donor orbital and the receptor orbital for each of the structures was investigated using the natural bond orbital analysis. NBO analysis aids in the translation of computational solutions of Schrodinger's wave equations.^50,51^ It is an effective tool for interpreting the hyper-conjugative interactions and delocalization of electron density within the studied structures. It also provides information on the type of bonding and the nature of interactions present in the valence space between the virtual and occupied Lewis orbitals. The intensity of the donor–receptor interaction was denoted by the second-order stabilization energy, *E*^2^ (kcal mol^−1^). Large values of *E*^2^ indicate a strong interaction between donor orbitals (*i*) and the receptor orbitals (*j*) and express a more donating tendency from an electron donor to an electron receptor and accordingly a higher degree of conjugation of the whole system.^52–54^ The stabilization energy, *E*^2^ could be determined using eqn (5);5where *q*_*i*_ = donor orbitals occupancy; *E*(*j*) − *E*(*i*) = diagonal element; *F*(*i*, *j*) = off diagonal NBO Fock matrix element.^55^

From Table S2,† it is observed that the interaction which gave the highest stabilization energy result from π* → π*, LP → π*, LP → LP*, π → π*, π → LP*, LP → σ*, π* → σ*, σ → σ*, and σ → π*. Although these were not the only interactions that occurred in our studied systems, other interactions like RY (Rydberg) and Cr (centre core pair) where loosely bond interactions occur were also observed. The prominent intramolecular hyper-conjugative interactions resulted in the highest stabilization of 62.43 and 37.35 kcal mol^−1^ energy corresponding to π*(N_4_–C_5_) → π*(C_7_–C_8_) and π*(C_1_–O_2_) → π*(C_12_–C_16_) respectively, for L_1_ while those for L_2_ were 71.32, 33.17, and 32.15 kcal mol^−1^ corresponding to π*(C_1_–O_2_) → π*(C_12_–C_16_), LP(2) S_11_ → π*(C_7_–C_8_), and LP(2) S_13_ → π*(C_14_–C_15_) respectively. The highest stabilization energy of L_3_ as observed from the NBO analysis was 44.01 kcal mol^−1^ for the donor–acceptor interaction from π*(C_1_–O_2_) → π*(C_12_–C_16_), and 33.20 kcal mol^−1^ for LP(2) S_11_ → π*(C_7_–C_8_), while the highest *E*^2^ values for L_4_ were 121.46, 67.78, and 66.07 kcal mol^−1^, which correspond to the interaction between π*(C_9_–C_10_) → π*(C_7_–C_8_), LP(2) N_22_ → π*(C_12_–C_13_), and π*(C_1_–O_2_) → π*(C_11_–C_14_). For the L_1_Ni complex, the highest stabilization energies resulting from the donor–acceptor interactions were observed to be 41.69, and 20.47 kcal mol^−1^ arising from the interaction of π(C_7_–C_13_) → π*(O_2_–C_6_), and LP(2) O_2_ → LP*(6) Ni_45_, respectively; for L_2_Ni, it was observed from π*(C_35_–C_41_) → π*(C_36_–C_37_) with an *E*^2^ of 66.79 kcal mol^−1^, π*(C_7_–C_13_) → π*(C_8_–C_9_) with an *E*^2^ of 57.27 kcal mol^−1^, and LP(1) N_4_ → LP*(6) Ni_47_, with stabilization energies of 22.78 kcal mol^−1^, respectively. The L_3_Ni complex has its most significant interaction resulting in the stability of the system from π*(C_7_–C_13_) → π*(C_8_–C_9_) and π(C_7_–C_13_) → π*(O_2_–C_6_) with stabilization energies of 56.34 and 41.09 kcal mol^−1^, respectively, L_4_Ni also had it most significant interaction resulting in the stability of the system from π(C_18_–C_19_) → LP*(2) N_46_ and π*(C_17_–C_23_) → π*(C_18_–C_19_) with stabilization energy of 92.86 and 51.01 kcal mol^−1^ respectively. L_1_Ni on adsorption of H_2_S had its strongest interaction from LP(2) O_25_ → σ*(C_9_–H_12_) and π*(C_18_–C_24_) → σ*(C_9_–H_12_) which gave an *E*^2^ value of 1227.96 and 1211.30 kcal mol^−1^ respectively, while L_2_Ni–H_2_S had it highest *E*^2^ value from σ(C_36_–C_37_) → π*(C_25_–C_46_) and σ(C_18_–H_21_) → σ*(C_19_–H_22_) corresponding to 15 641.30 and 7484.17 kcal mol^−1^ respectively. For L_3_Ni–H_2_S, the highest stabilization energy resulted from the interactions of σ(N_5_–H_14_) → σ*(C_36_–H_39_) and LP(1) S_48_ → σ*(C_9_–H_12_) corresponding to 5278.79 and 2093.84 kcal mol^−1^ respectively; also L_4_Ni–H_2_S showed it highest stabilization energy from the interaction of σ(S_48_–H_49_) → σ*(C_33_–C_41_) and LP(1) S_48_ → σ*(S_48_–H_50_) which correspond to 8244.44 and 7726.42 kcal mol^−1^. This result suggests that the stability of our complex on H_2_S adsorption is in the order L_2_Ni–H_2_S > L_4_Ni–H_2_S > L_3_Ni–H_2_S > L_1_Ni–H_2_S based on the stabilization energy values since it has been asserted that the higher the stabilization energy, the greater the interaction and the higher the overall stability of the system. From the above discussion, it is evidently concluded that the designed systems are good candidates for efficient H_2_S adsorption.

### 3.7 Density of state

The density of state (DOS) is an important parameter in solid physics which reveals the number of states in unit energy interval for a given chemical system. Its graph is used for analyzing the nature of electron structure along with the distribution of molecular orbitals with their associated energies. In this work, we employed the Multiwfn software for the calculation of the DOS of the studied compounds. The comparison between the DOS plots of L_1_Ni, L_2_Ni, L_3_Ni and L_4_Ni *versus* that of their interaction with H_2_S demonstrated the changes in the electronic properties of the complexes upon the adsorption process that can be used to determine the sensitivity of the stated complexes towards H_2_S. Upon interaction of each complex with H_2_S, it can be concluded that some new energy states appeared around the Fermi level (*E*_FL_) which resulted to an increase in the *E*_g_ values. The difference in the *E*_g_ was calculated as 0.1347, 0.1474, 0.1435, and 0.1704 eV for L_1_Ni–H_2_S, L_2_Ni–H_2_S, L_3_Ni–H_2_S and L_4_Ni–H_2_S, respectively. It can be concluded that the maximum and minimum alterations in the *E*_g_ were observed for L_4_Ni–H_2_S and L_1_Ni–H_2_S respectively (Fig. 5).

**Fig. 5:** Projected density of states for the complexes and H_2_S adsorbed complexes.

### 3.8 Topological analysis

In this study QTAIM and NCI were employed as topological analysis to vividly study the kinds of intermolecular interaction of the investigated surfaces and the adsorption characteristic behaviors of L_1_Ni, L_2_Ni, L_3_Ni and L_4_Ni for H_2_S.

#### 3.8.1 Quantum theory of atoms-in-molecules (QTAIM)

The quantum theory of atoms-in-molecules proposed by Richard F. W. Bader and colleagues^42^ was used to further analyze the type and structure of bonds and intermolecular interactions using topological parameters such as total electronic density (*ρ*), Laplacian of electron densities (*∇*^2^*ρ*), Lagrangian kinetic energy *G*(*r*), Hamiltonian kinetic energy *K*(*r*), total electronic energy *H*(*r*), potential energy (*V*), electron localization function (ELF) and ellipticity (*ε*) at the bond critical point (BCP). A bond critical point is a saddle point between two bonded atoms in which there is a maximum distribution of electron density. The BCP is useful in characterizing different types of interaction existing between the bond path of two bonded atoms. Table 4 shows the calculated topological parameters for the complex and its interaction with H_2_S. One of the most significant relationships between topological parameters is given by eqn (6) and (7) at a CPs (critical point):6

7 *H*(*r*) = −*K*(*r*)

**Table 4:** The calculated topological parameters: electron density *ρ*(*r*), Laplacian electron density *∇*^2^*ρ*(*r*), Lagrangian kinetic energy *G*(*r*), Hamiltonian kinetic energy *K*(*r*), potential electron energy density *V*(*r*), total electron energy density *H*(*r*), |*V*(*r*)|/*G*(*r*) ratio at the bond critical points (BCPs), ellipticity (*ε*), electron localization function (ELF), and eigenvalues (*λ*_1_, *λ*_2_, *λ*_3_) for the optimized complexes before and after adsorption of H_2_S gas. All the values are in a.u.

Interaction	BCP	*ρ*(*r*)	*∇* ^2^ *ρ*(*r*)	*G*(*r*)	*K*(*r*)	*V*(*r*)	*H*(*r*)	|*V*(*r*)|/*G*(*r*)	*ε*	ELF	*λ*_1_	*λ*_2_	*λ*_3_
**L**_**1**_ **Ni**													
Ni_45_–O_2_	67	0.1103	0.7201	0.1981	0.0181	0.2162	−0.0181	1.0914	0.1896	0.1191	−0.1421	−0.1691	1.0313
C_26_–N_33_	76	0.3310	−0.9693	0.2126	0.4550	−0.6676	−0.4550	3.1402	0.1834	0.8206	−0.7693	0.4501	−0.6501
Ni_45_–N_4_	82	0.0966	0.4414	0.1329	0.0225	−0.1554	−0.0225	1.1693	0.0934	0.1618	−0.1087	−0.1188	0.6689
C_16_–N_1_	85	0.3701	−0.8832	0.3323	0.5531	−0.8853	−0.5531	2.6642	0.2344	0.7311	0.6186	−0.8297	−0.6721

**L**_**2**_ **Ni**													
C_35_–H_38_	52	0.2911	−1.0846	0.0309	0.3020	−0.3329	−0.3020	10.7735	0.0291	0.9930	0.6504	−0.8799	−0.8550
Ni_47_–N_4_	80	0.0967	0.4409	0.1330	0.0227	−0.1557	−0.0227	1.1707	0.0798	0.1622	−0.1098	−0.1186	0.6693
Ni_47_–O_2_	92	0.1103	0.7187	0.1979	0.0182	−0.2161	−0.0182	1.0920	0.1766	0.1194	−0.1430	−0.1682	1.0299
O_2_–C_6_	96	0.3703	0.4475	0.5924	0.5812	−1.1736	−0.5812	1.9811	0.0199	0.4613	1.9480	−0.9422	−0.9610

**L**_**3**_ **Ni**													
Ni_47_–N_4_	62	0.6709	0.2327	0.4884	−0.9327	−0.3952	0.9327	1.2358	0.1924	0.0956	0.3292	−0.5048	−0.4607
Ni_47_–O_2_	79	0.3508	0.1375	0.3369	−0.6685	−0.3303	0.6685	1.0200	0.9301	0.0256	0.2480	−0.547	−0.5610
Ni_47_–O_3_	85	0.3068	−0.1457	0.3589	0.4002	−0.1899	−0.4002	1.8899	0.9920	0.0275	−0.1319	0.1145	−0.1283
Ni_47_–N_1_	94	0.3492	0.2541	0.1641	0.1714	−0.1812	−0.1714	0.9056	0.8569	0.0593	0.3597	−0.5431	−0.5127

**L**_**4**_ **Ni**													
Ni_47_–N_4_	72	0.0886	0.4803	0.1339	0.0138	−0.1477	−0.0138	1.1031	0.1378	0.1248	−0.0511	−0.0581	0.5895
Ni_47_–O_2_	79	0.0939	0.6089	0.1612	0.0089	−0.1701	−0.0089	1.0552	0.5117	0.1067	0.8430	−0.0932	−0.1409
Ni_47_–O_3_	85	0.0931	0.5907	0.1566	0.0089	−0.1655	−0.0089	1.0568	0.5217	0.1094	0.8288	−0.0944	−0.1437
Ni_47_–N_1_	92	0.0896	0.4796	0.1344	0.0145	−0.1488	−0.0145	1.1071	0.1618	0.1281	−0.0552	0.5989	−0.0641

**L**_**1**_ **Ni–H**_**2**_ **S**													
S_48_–H_17_	69	0.0107	0.0337	0.0070	−0.0015	−0.0055	0.0015	0.7857	0.2881	0.0434	0.0506	−0.0074	−0.0095
Ni_45_–S_48_	80	0.0282	0.0374	0.0152	0.0058	−0.0210	−0.0058	1.3816	0.2345	0.1972	−0.0173	0.0760	−0.0213
Ni_45_–N_1_	89	0.0802	0.3630	0.1047	0.0139	−0.1186	−0.0139	1.1328	0.6289	0.1431	0.5309	−0.0639	−0.1040
Ni_45_–O_3_	96	0.0980	0.6287	0.1680	0.0109	−0.1789	−0.0109	1.0649	0.3452	0.1123	0.8778	−0.1062	−0.1429

**L**_**2**_ **Ni–H**_**2**_ **S**													
S_48_–H_16_	68	0.0112	0.0350	0.0072	−0.0015	−0.0057	0.0015	0.7917	0.2672	0.0469	0.0530	−0.0079	−0.0101
Ni_47_–S_48_	81	0.0278	0.0371	0.0149	0.0057	−0.0206	−0.0057	1.3826	0.2335	0.1939	−0.0168	0.0746	−0.0207
Ni_47_–N_1_	89	0.0836	0.3790	0.1100	0.0153	−0.1253	−0.0153	1.1391	0.5364	0.1482	0.5580	−0.0706	−0.1084
Ni_47_–O_3_	95	0.0973	0.6223	0.1663	0.0107	−0.1769	−0.0107	1.0637	0.3393	0.1122	0.8709	−0.1063	−0.1423

**L**_**3**_ **Ni–H**_**2**_ **S**													
S_48_–H_16_	66	0.0102	0.0324	0.0067	−0.0014	−0.5207	0.0014	77.7164	0.3059	0.4118	0.0481	−0.0068	−0.0089
Ni_47_–S_48_	80	0.0285	0.0374	0.0153	0.0059	−0.0212	−0.0059	1.3856	0.2252	0.1997	−0.0174	0.0762	−0.0214
Ni_47_–N_1_	88	0.0811	0.3694	0.1066	0.0142	−0.1208	−0.0142	1.1332	0.6158	0.1434	0.5397	−0.0651	−0.1052
Ni_47_–O_3_	93	0.0978	0.6231	0.1666	0.0109	−0.1775	−0.0109	1.0654	0.3627	0.1133	0.8755	−0.1068	−0.1456

**L**_**4**_ **Ni–H**_**2**_ **S**													
Ni_47_–S_48_	71	0.0368	0.0384	0.0193	0.0097	−0.0289	−0.0097	1.4974	1.4773	0.2696	−0.0179	−0.0443	0.1007
Ni_47_–N_4_	74	0.0907	0.4940	0.1382	0.0147	−0.1529	−0.0147	1.1064	0.0706	0.1265	−0.0558	−0.0597	0.6095
Ni_47_–O_2_	76	0.0962	0.6095	0.1626	0.0102	−0.1728	−0.0102	1.0627	0.4443	0.1130	0.8662	−0.1050	−0.1517
Ni_47_–N_1_	89	0.0923	0.4917	0.1387	0.0157	−0.1544	−0.0157	1.1132	0.1456	0.1321	−0.0611	0.6229	−0.0700

Based on the AIM theory, a positive value for total electronic energy density (*ρ*) at a BCP indicates closed shell interactions. When *∇*^2^*ρ* > 0 and *H* > 0 it indicative of a weak covalent interaction (strong electrostatic bond), while *∇*^2^*ρ* < 0 and *H* < 0 values denotes a strong covalent bond, and the *H* < 0 and *∇*^2^*ρ* > 0 denote the medium strength or partially covalent bond. According to the results given in Table 4, the *∇*^2^*ρ* values of the studied systems are positive whereas their *H*(*r*) values are mostly negative and this shows that the bond present in the studied system is composed of a partial covalent bond. Also according to literature review, if |*V*(*r*)|/*G*(*r*) < 2 but >1 then a mixed character interactions is present. If |*V*(*r*)|/*G*(*r*) > 2 it indicates covalent bonds and when |*V*(*r*)|/*G*(*r*) < 1 then it is indicative of the presence of ionic bonds and van der Waals interactions.^44^ The bond ellipticity, *ε*, is an important parameter used to predict the stability of interactions. High values of *ε* (*i.e.*, *ε* > 1) indicate structural instability, and lower values of *ε* indicate structural stability of the interactions (*i.e.*, *ε* < 1). The ellipticity values for our complexes before and after adsorption of H_2_S are in the range of 0.0199 to 1.4773 a.u. This result demonstrates that the bond in our studied compound is a sigma bond. Electron localization function (ELF) is also an important tool that is used to analyze covalent bonding. If the ELF value is between 0.5 and 1, it indicates regions containing bonding and non-bonding localized electron, when the value of ELF is lower than 0.5, it reveals that the electron is delocalized. From the values obtained in Table 4, for the complexes after the adsorption of H_2_S, it can be stated that the electrons are delocalized because their values are less than 0.5.

#### 3.8.2 Noncovalent interaction (NCI)

Multiwfn software^41^ was employed to analyze the noncovalent bonds. Non-covalent interaction emanates through a number of different mechanisms such as the van der Waals interactions, hydrogen bonding, and electrostatic interactions. The second density Hessian eigenvalue *λ*_2_(*r*), the electron density *ρ*(*r*) and reduced density gradient (RDG) are the basic functions present in NCI analysis for the prediction of weak interactions. Isosurface plots involving the two functions give information on the type of weak interaction present. In the isosurface plot, the reduced density gradient (RDG) is plotted against the second eigenvalue of the electron density Hessian matrix (*λ*_2_) and the electron density *ρ*(*r*) that is the NCI graph is a graph of RDG against *λ*_2_(*r*)*ρ*(*r*). From the isosurface, the nature of weak interaction can be characterized depending on the values of *λ*_2_. The blue region with negative values, *λ*_2_(*r*)*ρ*(*r*) < 0 corresponds to strong interactions (such as hydrogen bonding) and high electron density, while the red region with positive values (*λ*_2_(*r*)*ρ*(*r*) > 0) indicates a strong repulsive interaction (like steric effect) and electron density depletion; the green region (sign *λ*_2_(*r*)*ρ*(*r*) ≈ 0) corresponds to relatively weak van der Waal interactions.^56,57^ As evident from the plots in Fig. 6, the blue regions existing between H_2_S and the complexes indicate the presence of strong hydrogen-bonding interactions. The green region observed between the H_2_S and the complexes indicates that van der Waals interactions play a key role in the adsorption of the gas by the complexes. In addition, little repulsion interaction is observed during the adsorption process. These are in good agreement with the adsorption energy and the QTAIM results.

**Fig. 6:** Pictorial view of the noncovalent interaction of the studied systems.

### 3.9 Adsorption studies

In this section, the adsorption of H_2_S gas on L_1_Ni, L_2_Ni, L_3_Ni and L_4_Ni systems is investigated. Several orientations for the adsorption of H_2_S were investigated, and only the most energetic stable orientations have been illustrated (Fig. 7). Fig. 1 and 7 shows the optimized structures of L_1_Ni, L_2_Ni, L_3_Ni and L_4_Ni systems before and after H_2_S adsorption. The adsorption energies, adsorption distance, energy gap, and fraction of electron transfer of the four systems after H_2_S adsorption are given in Table 5. The energy gaps of the four systems before and after gas adsorption were investigated and the results are presented in Fig. 3, 4 and Table 3. The energy gap results show that the systems are all semi-conductors before and after the adsorption of H_2_S. It worth noting that after the adsorption of H_2_S that the energy gap of the four systems increased from 7.0148 eV to 7.1495 eV for L_1_Ni, 7.0328 eV to 7.1802 eV for L_2_Ni, 6.9721 eV to 7.1156 eV for L_3_Ni and 3.2498 eV to 3.4202 eV for L_4_Ni. As can be seen from the results obtained in Table 5, the *E*_ads_ values for all interaction are negative, this indicates that there is a strong interaction between the complexes and H_2_S^58^ and the type of adsorption that exist is chemisorption. Furthermore, the adsorption energies follow the trend L_3_Ni–H_2_S > L_1_Ni–H_2_S > L_2_Ni–H_2_S > L_4_Ni–H_2_S for all the investigated complexes.

**Fig. 7:** Optimized structure of the complex after adsorption of H_2_S.

**Table 5:** Adsorption energy (*E*_ads_), adsorption distance (*D*), energy gap (Δ*E*_g_) and fraction of electron transfer (Δ*N*) of the four systems after the adsorption of H_2_S gas calculated at ωB97XD/gen level of theory

Structures	*E*_ads_ (kcal mol^−1^)	*D* (Å)	Δ*E*_g_	Δ*N*
L_1_Ni–H_2_S	−36.9465	2.8900	7.1495	1.3821
L_2_Ni–H_2_S	−35.9883	2.8983	7.1802	1.3684
L_3_Ni–H_2_S	−37.3224	2.9016	7.1156	1.3800
L_4_Ni–H_2_S	−29.5626	2.7173	3.4202	3.1225

### 3.10 Sensing mechanism

Herein, our main purpose is to investigate the ability of the complexes in the detection of H_2_S gas. To elucidate the mechanism of the gas sensor, the resistance changes of the complexes with and without the adsorption of gas are evaluated. The sensitivity of the complexes could be determined by the change in the electrical resistance (*σ*) after and before gas adsorption and the sensing response (*S*) and they could be determined through eqn (8) and (9):89where *σ* is the electrical conductivity, *A* is the Richardson constant, *T* is the working temperature and *K* is the Boltzmann constant (8.318 × 10^−3^ kJ mol^−1^ K^−1^), *σ*_gas_ and *σ*_pure_ are the conductivity of the complex after and before adsorption. According to eqn (3), the electrical conductivity of the adsorbent increases as the *E*_g_ value decrease. From the results tabulated in Table 6, it can be seen that the *E*_g_ of the complexes is affected by the presence of H_2_S. It was discovered that the HOMO and LUMO values for all the complexes decreased after the adsorption of H_2_S which resulted in an increment in the energy gap values. For L_1_Ni the percentage increment in *E*_g_ after adsorption of H_2_S was calculated to be 1.92%, for L_2_Ni % Δ*E*_g_ was 2.10%, L_3_Ni has an increment of 2.06% and for L_4_Ni it was 5.24%. This substantial change in *E*_g_ after the adsorption process affects the electrical conductivity of the complexes as stated earlier with this change in the conductivity, the investigated complexes hold a prospect to detect H_2_S and from the findings of this study, L_1_Ni has a much better H_2_S detection followed by L_3_Ni then L_2_Ni and L_4_Ni. This implies that the sensing response for the complexes follows the order L_1_Ni > L_3_Ni > L_2_Ni > L_4_Ni.

**Table 6:** Calculated HOMO energies (*E*_HOMO_), LUMO energies (*E*_LUMO_), Fermi level energy (EF), HOMO–LUMO energy gap (*E*_g_), work function (*Φ*) and recovery time of the complexes after H_2_S adsorption. Energies are in eV. % Δ*E*_g_ and % Δ*Φ* indicate the change of *E*_g_ and work function after H_2_S adsorption, respectively

Structures	*E*_HOMO_	*E*_LUMO_	*E*_f_	*E*_g_	% Δ*E*_g_	*E*_ads_	*Φ*	% Δ*Φ*	*τ*
L_1_Ni	−13.8860	−6.8712	−10.3786	7.0148	−13.12	—	10.3786	149.44	—
L_2_Ni	−13.8182	−6.7854	−10.3018	7.0328	−12.68	—	10.3018	136.83	—
L_3_Ni	−13.7899	−6.8178	−10.3039	6.9721	−13.77	—	10.3039	139.10	—
L_4_Ni	−13.1205	−9.8707	−11.4956	3.2498	659.30	—	11.4956	296.21	—
L_1_Ni–H_2_S	−13.7943	−6.6448	−10.2196	7.1495	1.92	−36.9465	10.2196	−1.53	2.973 × 10^−6^
L_2_Ni–H_2_S	−13.7330	−6.5528	−10.1429	7.1802	2.10	−35.9883	10.1429	−2.27	2.02 × 10^−6^
L_3_Ni–H_2_S	−13.7048	−6.5892	−10.1470	7.1156	2.06	−37.3224	10.1470	−1.52	3.46 × 10^−6^
L_4_Ni–H_2_S	−13.0250	−9.6048	−11.3149	3.4202	5.24	−29.5626	11.3149	−1.57	1.511 × 10^−7^

The effect of H_2_S on the Fermi level (*E*_f_) and work function (*Φ*) are also investigated. The work function basically is the energy required to remove an electron from the Fermi level while the Fermi level which is the midpoint of the HOMO and LUMO energy gap. The quantitative value of change in the work function and Fermi level on the complexes due to the adsorption of the gas molecule can be evaluated through eqn (10) and (11):

10 *Φ* = *V*_el(+∞)_ − *E*_f_

11where, *V*_el(+∞)_ and *E*_f_ are the electrostatic potential energy of the electron far from the surface of the material which equals zero, and the energy of Fermi level of the sensing material. Where *V*_el(+∞)_ equals zero the work function is the negative of the Fermi level which is the midpoint of the HOMO and LUMO energy gap. It is worth noting that when the adsorption process changes the work function of the adsorbent, it influences the gate voltage, creating a noise which helps the gas detection.^59^Fig. 8 shows the variation in work function on adsorption of H_2_S on the complexes. The variation in work function after adsorption of the gas molecule describes the charge transfer among the two interacting entities. We have obtained the value of the work function for L_1_Ni, L_2_Ni, L_3_Ni, and L_4_Ni as 10.2196 eV, 10.1429 eV, 10.147 eV and 11.3249 eV respectively. From these values, it indicates that our complexes are highly affected by H_2_S. Based on the Richardson Dushman equation (eqn (12)), the electron current density emitted from the surface of the sensor (*j*) will be related to the work function (*Φ*) as follows:^60^

12 *j* = *AT*^2^e^(−*Φ*/*kT*)^

where *A* is called the Richardson constant (A m^−2^), *k* is the Boltzmann constant and *T* is the temperature (K). From Table 6 it is shown that the work function (*Φ*) value decreases for all the complexes on adsorption of H_2_S by 1.52%, 2.27%, 1.52%, and 1.57% for L_1_Ni, L_2_Ni, L_3_Ni, and L_4_Ni respectively. Consequently, the emitted electron current density from the surface of the complexes will decrease after the adsorption of H_2_S. The negative values of the adsorption indicate exothermic interactions which implies strong interaction. The strength of the adsorption affects the sensing mechanism of the systems because strong interactions between the adsorbent and the adsorbate indicate that desorption could be difficult and the device may suffer from long recovery times.

**Fig. 8:** Recovery time and work function of the complexes after adsorption of H_2_S.

The recovery time (*τ*), which is the time taken by the sensor to get back 80% of its original resistance is an indicator to evaluate the reproducibility of the gas sensor. A shorter recovery time indicates a better performance of the sensor material and it can be calculated using eqn (13)13where *A*, *T*, and *k* are the vibrational frequency (10^12^ s^−1^), temperature, and Boltzmann's constant, respectively. The calculated recovery time, *τ*, of H_2_S from the L_1_Ni, L_2_Ni, L_3_Ni, and L_4_Ni surfaces are 2.973 × 10^−6^ s, 2.02 × 10^−6^ s, 3.46 × 10^−6^ s, and 1.511 × 10^−7^ s respectively. This indicates that the complex senor benefits from a short recovery time.

### 3.11 Thermodynamic study

Thermodynamics is the study of the interaction of heat and work with chemical reactions or with physical changes of state within the confines of the law of thermodynamics. It is the application of mathematical methods to the study of chemical equations and the spontaneity of processes.^51,61^ Herein, we are concerned with the changes in Gibbs free energy, Δ*G* and enthalpy, Δ*H*. The enthalpy of a system is the sum of the system's internal energy, *Q* with the product of its pressure, *P* and volume, *V*, that is; Δ*H* = *Q* + *PV*. The enthalpy of a system may be positive or negative depending on whether heat is absorbed or evolved. When heat is absorbed by the system, Δ*H* is positive and the reaction is said to be endothermic, when heat is evolved by the system, Δ*H* is negative and the reaction is exothermic. On the other hand, the Gibbs free energy, Δ*G*, of a system is the change in its enthalpy, Δ*H* minus the product of the systems temperature, *T* and change in its entropy Δ*S*, that is, Δ*G* = Δ*H* − TΔS. The value of a system's Gibbs free energy gives information about the spontaneity of the system. If, Δ*G* < 0 the reaction is spontaneous, when Δ*G* > 0 the reaction is non-spontaneous and when Δ*G* = 0 the reaction is at equilibrium. When a reaction is at equilibrium, Δ*H* = *T*Δ*S* and this shows the system's tendency towards maximum entropy.

The calculation of the enthalpy and the Gibbs free energy of the reaction for the complexes under investigation was obtained from the optimized structures using eqn (14)–(17):

14 Δ*H*^0^(298 K) = Σproduct Δ_f_*H*^0^ prod.(298 K) − Σreactant Δ_f_*H*^0^ react.(298 K)

15 Δ_f_*H*^0^(298 K) = Σ(*ε*_0_ + *H*_Corr_) product − Σ(*ε*_0_ + *H*_Corr_) reactant

16 Δ*G*^0^(298 K) = Σproduct Δ_r_*G*^0^ prod.(298 K) − Σreactant Δ_r_*G*^0^ react.(298 K)

17 Δ_r_*G*^0^(298 K) = Σ(*ε*_0_ + *G*_Corr_) product − Σ(*ε*_0_ + *G*_Corr_) reactant

where *ε*_0_ is the electronic energy, *H*_Corr_ thermal correction to *H*, *G*_Corr_ thermal correction to *G*, Δ_f_*H*^0^ and Δ_f_*G*^0^ are the standard enthalpy and Gibbs free energy of formation for the products with other thermodynamic properties like zero-point energy (ZPE), constant volume, heat capacity, and entropy have been calculated at a constant temperature of 298.15 K using DFT methods. Table S3† shows detailed calculations of the enthalpy and free energy of the sensor material and the adsorbed gas. It can be deduced from the tabulated values for the enthalpy of formation which are 35.9821 kcal mol^−1^ for L_1_Ni, 35.6033 kcal mol^−1^, for L_2_Ni, 36.3453 kcal mol^−1^ for L_3_Ni, and 29.7615 kcal mol^−1^ for L_4_Ni that heat is absorbed when the complexes interact with H_2_S, that is, the reaction is endothermic since Δ_f_*H*^0^ is positive. Also, the calculated values of Δ_f_*G*^0^ for the complexes after H_2_S adsorption are 24.3477 kcal mol^−1^ for L_1_Ni, 23.4389 kcal mol^−1^ for L_2_Ni, 24.2133 kcal mol^−1^ for L_3_Ni, and 18.8009 kcal mol^−1^ for L_4_Ni. These values are also positive and indicate that the reaction is nonspontaneous.

## 4. Conclusions

The interaction of H_2_S gas with L_1_Ni, L_2_Ni, L_3_Ni and L_4_Ni was examined using appropriate DFT calculations with Gen/6-311+G(d,p)/LanL2dZ basis set using ωB97XD functional. Spectroscopic characterization, adsorption energy, natural bond orbital (NBO), frontier molecular orbital (FMO), the density of state (DOS), topological quantum theory of atom-in-molecule (QTAIM) analyses, thermodynamics, sensing mechanism, and non-covalent interaction (NCI) assessments were highlighted in this study. From the FMO calculations, L_4_Ni was observed to have the smallest energy gap of 3.2498 eV, which results in the highest conductivity and least stability. The most stable is L_2_Ni, which has the largest energy range of 7.0328 eV. The density of state (DOS) plot, shows the major contribution of the complexes with H_2_S. The NBO analyses invoke insight into the energy stabilization of the complexes on interactions with H_2_S. It is also worthy to note that stabilization further increased the adsorption of H_2_S. Hence, indicates and suggests that the complexes possessed better candidacy for H_2_S adsorption. More so, more studies await these scientific observations. Thus, the sensing mechanism of the complexes indicated that all of them to have a short recovery time and that the work function value increases for all of them, making them an excellent H_2_S sensor. However, the Q-TAIM analyses gave insight into the bond existing between the studied systems. Thus, a profound assertion was given that the complex sensor surfaces exhibited very dense stability with regards to their relevant binding energies corresponding to various existing studies. With respect to the adsorption energies of the systems, L_3_Ni–H_2_S has the maximum adsorption capacity. Notwithstanding, the thermodynamics study, the interaction of the complexes with H_2_S showed non-spontaneous thermodynamics properties.

## Data availability

All data are contained within the manuscript and ESI.†

## Author contributions

Hitler Louis: project conceptualization, design, and supervision. Daniel Etiese: writing, results extraction, analysis, and manuscript first draft. Tomsmith O. Unimuke: validation, visualization, manuscript revision, and editing. Aniekan E. Owen: resources, review, writing, and editing. Terkumbur E. Gber: manuscript review, and proofreading. Ededet A. Eno: manuscript proofreading. Abdullah O. Rajee: resources, review, and editing. Chioma Chima: data curation. Emmanuel N. Nfor: review and editing.

## Conflicts of interest

All authors declare zero financial or inter-personal conflict of interest that could have influenced the research work or results reported in this research paper.

## Supplementary Material

RA-012-D2RA05456F-s001
